The article "Nonlinear Dynamic Response Analysis of a Three-Stage Gear Train Based on Lightweight Calculation for Edge Equipment" was published in 2022. Journal: Comput Intell Neurosci.

# Nonlinear Dynamic Response Analysis of a Three-Stage Gear Train Based on Lightweight Calculation for Edge Equipment

**DOI:** 10.1155/2022/4724504

**Published:** 2022-08-21

**Authors:** Dongdong Ren, Yangwu Yao, Huiyuan Wang, Huixian Qu, Guoqiang Wang

**Affiliations:** College of Mechanical and Electrical Engineering, North University of China, Taiyuan 030051, China

## Abstract

Bevel gears are widely used in aerospace transmission systems as well as modern mechanical equipment. In order to meet the needs and development of aerospace, high-speed dynamic vehicles, and various defense special equipment, higher and higher requirements are made for the high precision and stability of gear transmission systems, as well as the prediction and control of noise and vibration. Considering the nonlinear factors such as comprehensive gear error and tooth side clearance, a dynamic model of the three-stage gear transmission system is established. The relevant physical parameters, geometric parameters, and load parameters in the gear system are considered random variables to obtain the stochastic vibration model. When the random part of the random parameters is much smaller than the deterministic part, the vibration differential equation is expanded into a first-order term at the mean of the random parameter vector according to the Taylor series expansion theorem, and the ordering equation is solved numerically. Based on the improved stochastic regression method, the nonlinear dynamic response analysis of the three-stage gear train is carried out. This results in a relatively stable system when the dimensionless excitation frequency is in the range of 0.716 to 0.86 and the magnitude of the dimensionless integral meshing error is < 1.089.

## 1. Introduction

Gearing systems are widely used in various types of machinery and equipment, and ensuring the smoothness and accuracy of the transmission process has always been the goal of industrial production [1]. With the development of wind turbine drive train power towards the megawatt level, the accuracy of the dynamic response analysis of the three-stage gearbox drive train model has been increasing. Therefore, the study of the coupled nonlinear dynamic characteristics of large generator gearboxes under variable loads, and then provide important theoretical value and practical engineering significance for the design of three-stage gearboxes [2]. In recent years, many domestic and foreign scholars have conducted in-depth studies on the performance research methods and dynamics models of three-stage gearbox drive systems, and have made certain achievements [3, 4, 5]. The coupled nonlinear dynamics model of the gear-rotor-bearing-box of a large three-stage gearbox with multi-stage planetary gearing was established under the combined effect of internal and external load excitation, and the vibration response analysis of the three-stage gearbox was carried out by using the modal superposition method. Reference [6] accurately modeled the gearbox drive train of a large wind turbine and studied its drive train under variable wind loads. Reference [7] established a bending-torsion coupled dynamics model of a megawatt-class wind turbine gearbox drive train and calculated the structural sketch of the three-stage gearbox drive train using the fourth-order Runge–Kutta method.

The article "Nonlinear Dynamic Response Analysis of a Three-Stage Gear Train Based on Lightweight Calculation for Edge Equipment" was published in 2022. Journal: Comput Intell Neurosci.

Wind turbine gearboxes can be configured in different types, such as three-stage fixed shaft gear systems, planetary gear systems, and planetary and parallel shaft gear systems. The form of transmission mechanism used in the three-stage gearbox depends on the capacity requirements of the three-stage unit. The development of offshore three-stage technology and the need to reduce the cost of three-stage have strongly promoted the development of large single-capacity three-stage units. Three-stage planetary gearboxes are widely used in high-power double-fed three-stage gearboxes because of their strong load-bearing capacity, large speed increase ratio, and compact structure. Compared with single-stage planetary gearboxes, three-stage planetary gearboxes are more susceptible to vibration and noise and failure due to interstage coupling and three-stage transmission of torque [8]. Therefore, it is important to analyze the dynamic characteristics of three-stage planetary gear trains. A series of research results have been obtained for the analysis of the dynamics of a three-stage planetary gear train in three-stage gearboxes.

The dynamics of a single pair of a gear pair system has been studied more systematically. In [8], a time-varying nonlinear dynamics model was established, and the effect of side clearance on the meshing state and its frequency response characteristics was considered [9]. The parameters of the single-stage spur gear system are studied in detail, and the effects of parameter variations on the dynamic characteristics are presented. In [10], an approximate analytical solution of the three-stage nonlinear gear train was carried out using the harmonic balance method, and the effect of the variation of key parameters on the system response was analyzed [11]. The dynamic simulation technique of a three-stage gear train considering only the time-varying meshing stiffness was studied [12]. The nonlinearities of the intermediate shaft system and the idler system with time-varying meshing stiffness are investigated, and the analytical and numerical solutions are compared. In [13], the dynamic characteristics of the three-stage idler system with nonlinear parameter excitation are presented, and the periodic steady-state solutions are obtained by both analytical and numerical methods.

The article "Nonlinear Dynamic Response Analysis of a Three-Stage Gear Train Based on Lightweight Calculation for Edge Equipment" was published in 2022. Journal: Comput Intell Neurosci.

Tooth surface errors are unavoidable in the gear manufacturing process. In this paper, a modified stochastic regression method is used to solve the system of vibration differential equations for a three-stage gear train, and the effects of the changes of the integrated dimensionless excitation frequency and the integrated meshing error on the dynamic response of the system are analyzed. It is found that the system is in a relatively stable state when the dimensionless excitation frequency is in the range of 0.716–0.86 and the magnitude of the integrated dimensionless meshing error is <1.089.

## 2. Related Work

In order to meet the practical needs of low speed and a heavy load and a large transmission ratio, the study of the dynamics of the gear transmission system is becoming a hot spot for engineering applications and academic research. According to the research focus, [14] used the finite element method, the centralized parameter method, and the experimental modal analysis method, respectively. In [15], the finite element model and the centralized parametric model of the gear set were established, and the results of the two models were compared and analyzed, and the results of the two models were found to be consistent. In [16], the dynamic characteristics of the system under different fixation methods of the solar wheel were analyzed. In [17], the vibration model of the planetary gear was developed by the centralized parameter method considering the meshing phase relationship, and the modalities and vibration modes of the system were calculated for different modalities. In terms of nonlinear dynamics of planetary gear sets, [18] analyzed the dynamics of planetary gears under changing meshing stiffness by using rectangular waves to represent the time-varying meshing stiffness of the gear teeth. In [19], the effect of manufacturing errors on the nonlinear dynamics of planetary gears were studied, and the differences in the dynamics of the system under normal conditions, in the presence of tooth profile errors, and when centrifugal forces were considered and compared. In [20], the dynamics of planetary gears under strong nonlinear factors with multiple clearances is considered, and it is important to note that the analytical solution of the system vibration differential equations is obtained by the harmonic balance method, which is a typical application of the approximate analytical solution method under strong nonlinear factors. The study of the concentrated mass model of planetary gear sets focuses on the pure torsional vibration model and the meshing coupling model. Theoretical tooth surface and real tooth surface STE are introduced into the dynamics model in the form of discrete points, and the effects of real tooth surface STE and theoretical tooth surface STE on the dynamics performance of the curved bevel gear pair are compared and analyzed.

The article "Nonlinear Dynamic Response Analysis of a Three-Stage Gear Train Based on Lightweight Calculation for Edge Equipment" was published in 2022. Journal: Comput Intell Neurosci.

## 3. Complex Modal Structural Systems

The basic equation for the vibration of a gear system and the complex modal forced vibration equation for an N-dimensional linear system can be expressed as

(1) $$\begin{array}{c} M\ddot{X}+C\dot{X}+KX=Q\left(t\right), \end{array}$$

where *M*, *C*, and *K* denote the *N* ×*N* order mass matrix, damping matrix, and stiffness matrix, respectively, *X* and *Q*(*t*) denote the generalized displacement vector and external excitation, respectively, $M\ddot{X}$ denotes the generalized velocity vector and $C\dot{X}$ denotes the generalized acceleration vector. The free vibration equation of the complex modal structural system can be expressed as

(2) $$\begin{array}{c} M\ddot{X}+C\dot{X}+KX=0. \end{array}$$

It may be assumed that, *X*=*xe*^*λt*^ by substituting into (2), the corresponding right eigenvalue problem is obtained as follows:

(3) $$\begin{array}{c} \left(M\lambda^{2}+C\lambda +K\right)x=0. \end{array}$$

The corresponding concomitant eigenvalue problem is (*Mλ*^2^+*Cλ*+*K*)^*T*^*y*=0, and the left eigenvalue equation is obtained by transposing the concomitant eigenvalue equation as follows:

(4) $$\begin{array}{c} y^{T}\left(M\lambda^{2}+C\lambda +K\right)=0, \end{array}$$

where the vectors *x* and *y* denote the right and left eigenvalues, respectively, and *λ* denotes the eigenvalue of the vibration equation.

To simplify the above representation, a right state vector *u* is introduced to replace *x*, satisfying *u*=*λx*/*x*=*Tx*, where *T* is the state transition matrix and can be expressed as *T*=*λI*/*I*. Similarly, another left state vector *v* is used instead of *y*, satisfying *V*=*λY*/*Y*. Thus, (3) and (4) can be rewritten as

(5) $$\begin{array}{c} \left(A\lambda +B\right)u=0,\\ v^{T}\left(A\lambda +B\right)=0. \end{array}$$

Among them

(6) $$\begin{array}{c} A=\left[\begin{array}{cc} 0 & M\\ M & C \end{array}\right],B=\left[\begin{array}{cc} -M & 0\\ 0 & K \end{array}\right]. \end{array}$$

After the state transformation, (6) can be rewritten as

(7) $$\begin{array}{c} \left(A\lambda +B\right)u=0. \end{array}$$

(8) $$\begin{array}{c} v^{T}\left(A\lambda +B\right)=0. \end{array}$$

(7) and (8) have the same eigenvalues and can be derived from the following equation:

(9) $$\begin{array}{c} \det\left(A\lambda +B\right)=0. \end{array}$$

(8) is an algebraic equation with 2N eigenvalues in the complex domain, which can be expressed as *λ*_*i*_(*i*=1,2,…, *N*).

The article "Nonlinear Dynamic Response Analysis of a Three-Stage Gear Train Based on Lightweight Calculation for Edge Equipment" was published in 2022. Journal: Comput Intell Neurosci.

A and B can be expressed as

(10) $$\begin{array}{c} \left\{\begin{array}{c} A=A_{0}+\varepsilon A_{1}\text{,}\\ B=B_{0}+\varepsilon B_{1}\text{.} \end{array}\right.. \end{array}$$

## 4. Matrix Ingestion Method for Complex Modal Structural Vibrations

Since the non-diagonal of the consistent mass matrix contains non-zero elements, when vectorial finite elements are used for dynamic analysis, the consistent mass matrix is often replaced by the concentrated mass matrix in order to reduce computational effort and storage space. The most common method of constructing a centralized mass matrix is to distribute the mass of a cell equally among the connected nodes. When the mass of the unit or the internal nodes are not uniformly distributed, a higher-order difference function is used for mass distribution.

For the rod system structure, the elements on the main diagonal of each row of the centralized mass matrix element on each row of the consistent mass matrix is the sum of all elements in the corresponding row of the consistent mass matrix, i.e.,

(11) $$\begin{array}{c} M_{1}^{e}=diag\left(M_{c}^{e}\cdot J_{n}\right), \end{array}$$

where _*M*_^1^ is the concentrated mass matrix. _*M*_^*c*^ is the consistent mass matrix. *J*_*n*_ is the *n*th-order square matrix composed of 1. Substituting equation (5) into (6) further simplification yields

(12) $$\begin{array}{c} M_{1}=\left(\frac{1}{2}\right)diag\left(C^{T}\hat{m}C\right)⊗I_{3}. \end{array}$$

In practical engineering, the variation of structural parameters is reflected in the variation of the mass matrix. Considering the small perturbations of the parameters around their mean values, the mass matrix can be expressed as

(13) $$\begin{array}{c} \left\{M=M_{0}+\varepsilon M_{1}\right.,\\ \left\{C=C_{0}+\varepsilon C_{1}\right.\\ K=K_{0}+\varepsilon K_{1}. \end{array}$$

According to the matrix regression method, the eigenvalues and eigenvectors of a complex modal structural vibration system can be expanded into the form of a regression series:

(14) $$\begin{array}{c} \left\{\lambda^{i}\right.=\lambda_{0}^{i}+\varepsilon \lambda_{1}^{i}+\varepsilon^{2}\lambda_{2}^{i}+\cdots u^{i}\\ =u_{0}^{i}+\varepsilon u_{1}^{i}+\varepsilon^{2}u_{2}^{i}+\cdots \left\{v^{i}\right.\\ =v_{0}^{i}+\varepsilon v_{1}^{i}+\varepsilon^{2}v_{2}^{i}+\cdots x^{i}\\ =x_{0}^{i}+\varepsilon x_{1}^{i}+\varepsilon^{2}x_{2}^{i}+\cdots y^{i}\\ =y_{0}^{i}+\varepsilon y_{1}^{i}+\varepsilon^{2}y_{2}^{i}+\cdots \text{.} \end{array}$$

Substituting (11) and (13) into (12), we get

(15) $$\begin{array}{c} \left(A_{0}+\varepsilon A_{1}\right)\left(\lambda_{0}^{i}+\varepsilon \lambda_{1}^{i}+\varepsilon^{2}\lambda_{2}^{i}+\cdots \right)\\ +\left(B_{0}+\varepsilon B_{1}\right)\left(u_{0}^{i}+\varepsilon u_{1}^{i}+\varepsilon^{2}u_{2}^{i}+\cdots \right)=0. \end{array}$$

Similarly, substituting equations (12) and (13) into (14) gives

(16) $$\begin{array}{c} {\left(v_{0}^{i}+\varepsilon v_{1}^{i}+\varepsilon^{2}v_{2}^{i}+\cdots \right)}^{T}\left(\begin{array}{c} \left(A_{0}+\varepsilon A_{1}\right)\\ \left(\lambda_{0}^{i}+\varepsilon \lambda_{1}^{i}+\right. \end{array}\right.\left.\left.\varepsilon^{2}\lambda_{2}^{i}+\cdots \right)+\left(B_{0}+\varepsilon B_{1}\right)\right)=0. \end{array}$$

Expanding (15) and ignoring the terms of O(*ε*^2^), comparing the coefficients of the same power of *ε* on the left and right sides of the equation yields

(17) $$\begin{array}{c} \varepsilon^{0}:\left(A_{0}\lambda_{0}^{i}+B_{0}\right)u_{0}^{i}=0\text{,}\\ \varepsilon^{1}:\left(B_{0}+\lambda_{0}^{i}A_{0}\right)u_{1}^{i}+B_{1}u_{0}^{i}+\lambda_{0}^{i}A_{1}u_{o}^{i}+\lambda_{1}^{i}A_{0}u_{o}^{i}=0\text{,}\\ \varepsilon^{2}:\left(B_{0}+\lambda_{0}^{i}A_{0}\right)u_{2}^{i}+\left(B_{1}+\lambda_{0}^{i}A_{1}\right)u_{1}^{i}+\lambda_{1}^{i}A_{0}u_{1}^{i}+\lambda_{1}^{i}A_{1}u_{0}^{i}+\lambda_{2}^{i}A_{0}u_{0}^{i}=0\text{,} \end{array}$$

where *ε* is a small parameter and has *ε* = 0 for the original system; M_0_,C_0_,K_0_ denotes the mean values; and *ε*M_1_, *ε*C_1_, *ε*K_1_ denotes the first-order regression term of M_0_,C_0_,K_0_, respectively. Further, the same operation of (13) and (14) for (17) gives

(18) $$\begin{array}{c} \varepsilon^{0}:\left(\begin{array}{c} A\\ 0 \end{array}+B_{0}\right)Tv_{0}^{i}=0,\\ \varepsilon^{1}:\left(\begin{array}{c} B\\ 0 \end{array}+A_{0}\right)Tv_{1}^{i}+\left(\begin{array}{c} B\\ 1 \end{array}+A_{1}+A_{0}\right)Tv_{o}^{i}=0,\\ \varepsilon^{2}:\left(\begin{array}{c} B\\ 0 \end{array}+A_{0}\right)Tv_{2}^{i}+\left(\begin{array}{c} B\\ 1 \end{array}+A_{1}\right)Tv_{1}^{i}+\lambda_{1}^{i}A_{0}{}^{T}v_{1}^{i}+\lambda_{1}^{i}A_{1}{}^{T}v_{0}^{i}+\lambda_{2}^{i}A_{0}^{T}v_{0}^{i}=0, \end{array}$$

where *λ*_1_^*i*^ and *λ*_2_^*i*^ represent the first-order and second-order registers of the *i*th eigenvalue, respectively. In addition, the first-order and second-order registers of the left eigenvector and the first-order and second-order registers of the right eigenvector can also be found by (15).

The article "Nonlinear Dynamic Response Analysis of a Three-Stage Gear Train Based on Lightweight Calculation for Edge Equipment" was published in 2022. Journal: Comput Intell Neurosci.

Expanding *u*_1_^*i*^ on the original right state eigenvector *u*_0_^*s*^ yields

(19) $$\begin{array}{c} u_{1}^{i}=\sum_{s=1}^{2N}h_{is}^{1}u_{0}^{s}. \end{array}$$

Substituting (17) into (18) yields

(20) $$\begin{array}{c} \left(B_{0}+\lambda_{0}^{i}A_{0}\right)\sum_{s=1}^{2N}h_{is}^{1}u_{0}^{s}+\left(B_{1}+\lambda_{0}^{i}A_{1}\right)u_{0}^{i}+\lambda_{1}^{i}A_{0}u_{0}^{i}=0. \end{array}$$

The left multiplication of (19) by *v*_0_^*sT*^ has

(21) $$\begin{array}{c} v_{0}^{sT}\left(B_{0}+\lambda_{0}^{i}A_{0}\right)\sum_{s=1}^{2N}h_{is}^{1}u_{0}^{s}+v_{0}^{sT}\left(B_{1}+\lambda_{0}^{i}A_{1}\right)\\ u_{0}^{i}+v_{0}^{sT}A_{0}u_{0}^{i}\lambda_{1}^{i}=0. \end{array}$$

Considering the modal orthogonal normalization conditions expressed in (14) and (15), (20) can be reduced to

(22) $$\begin{array}{c} h_{is}^{1}\left(\lambda_{0}^{i}-\lambda_{0}^{s}\right)+v_{0}^{sT}\left(B_{1}+\lambda_{0}^{i}A_{1}\right)u_{0}^{i}+\lambda_{1}^{i}\delta_{is}=0. \end{array}$$

Only if *s*=*i*, then *λ*_0_^*i*^=*λ*_0_^*s*^ can be obtained from (22)

(23) $$\begin{array}{c} \lambda_{1}^{i}=-v_{0}^{iT}\left(B_{1}+\lambda_{0}^{i}A_{1}\right)u_{0}^{i}. \end{array}$$

(20) can be further rewritten as

(24) $$\begin{array}{c} \lambda_{1}^{i}=-y_{0}^{iT}\left({\left(\lambda_{0}^{i}\right)}^{2}M_{1}+\lambda_{0}^{i}C_{1}+K_{1}\right)x_{0}^{i}. \end{array}$$

## 5. Uncertainty Propagation Analysis of Random Complex Eigenvalues

The mass matrix, damping matrix, and stiffness matrix of real engineering structures are generally considered as stochastic structural parameters due to the variation of raw material properties of gears, manufacturing errors, and loading environment. In this paper, the matrix regression method is introduced to the eigenvalue analysis of complex modal structures with stochastic parameters, and also provides a basis for uncertainty propagation analysis of asymmetric systems. Considering the stochastic nature of the structural parameters, the stiffness matrix K, the mass matrix *M*, the damping matrix C, the complex eigenvalues *λ*_*i*_, the left complex eigenvector *y*, and the right complex eigenvector *x* can be expressed in the following form:

(25) $$\begin{array}{c} \left\{\begin{array}{c} K=K_{d}+\varepsilon K_{r},M=M_{d}+\varepsilon M_{r},C=C_{d}+\varepsilon C_{r},A=A_{d}+\varepsilon A_{r},\\ B=B_{d}+\varepsilon B_{r},\lambda^{i}=\lambda_{d}^{i}+\varepsilon \lambda_{r}^{i},y^{i}=y_{d}^{i}+\varepsilon y_{r}^{i},x^{i}=x_{d}^{i}+\varepsilon x_{r}^{i}, \end{array}\right. \end{array}$$

where *ε* is a small parameter, *K*_*d*_, *M*_*d*_, *C*_*d*_, *A*_*d*_, *B*_*d*_, *λ*_*d*_^*i*^, *λ*_*d*_^*i*^, *x*_*d*_^*i*^ and *K*_*r*_, *M*_*r*_, *C*_*r*_, *A*_*r*_, *B*_*r*_, *λ*_*r*_^*i*^, *y*_*r*_^*i*^, *x*_*r*_^*i*^ are the deterministic and random components of K, *M*, C, and *A*, *B*, *λ*^*i*^, *y*^*i*^, *x*^*i*^, respectively. Also, it is assumed that the mean value of *K*_*r*_, *M*_*r*_, *C*_*r*_, *A*_*r*_, *B*_*r*_, *λ*_*r*_^*i*^, *y*_*r*_^*i*^, *x*_*r*_^*i*^ is zero.

The article "Nonlinear Dynamic Response Analysis of a Three-Stage Gear Train Based on Lightweight Calculation for Edge Equipment" was published in 2022. Journal: Comput Intell Neurosci.

## 6. Numerical Solution of the Model

In this paper, we solve the differential equations of the system in terms of the magnitudes and vibrations, and briefly compare the results of the two numerical integration methods. Given the initial values of the system vibration, the first 800 transient response periods are omitted, and the dynamic response of the system is programmed in MATLAB to analyze the effect of the variation of excitation frequency, mesh damping ratio, and tooth side clearance on the bifurcation characteristics of the system. The basic parameters of the two-stage planetary gear train of the three-stage gearbox are as follows: rated power *P* = 2500 kW, normal speed range 16r/min∼21r/min, transmission ratio *i*_1_  = 5.25, *i*_2_  = 5.28, number of teeth of the first stage Zs = 31, Zpi = 47, Zr = 125, number of planetary wheels *N*_1_  =  *N*_2_  = 3, and the basic parameters of each gear are shown in Table 1.

The presence of static transmission error can aggravate the meshing shock of the gear teeth and cause abnormal vibration of the system, therefore, this paper discusses the effect of the integrated meshing error on the bifurcation characteristics of the system.

The kinetic analysis of the solution results by the global bifurcation diagram and maximum Lyapunov exponent (LLE) is shown in Figures 1 and 2. Given the dimensionless excitation frequency Ω_*m*_^1^  = 0.86, the mesh damping ratio *ξ* = 0.07 and the tooth side clearance *b* = 1, the effect of the integrated meshing error on the dynamic characteristics of the system is discussed with the dimensionless integrated meshing error magnitude *E* as the bifurcation parameter (for simplicity, the image coordinates *x*_*spi*_^(1)^ are denoted as _*x*_^*spi*^ and *E*_*spi*_^(1)^= as *E*). According to Figure 1, the three-stage planetary gear system has a rich nonlinear dynamic behavior when the magnitude of the integrated dimensionless meshing error is used as the bifurcation parameter. Combined with Figure 2, it is found that the system is relatively stable at low values of the integrated meshing error, when LLE is negative, and it is clear that the system enters the chaotic response as a multiperiodic bifurcation.

The dynamics of the two-stage planetary gear and the one-stage parallel shaft gear system are further verified and analyzed by combining the phase trajectory diagram and the Poncelet cross section diagram with the aid of the time history diagram and the spectrum diagram, as shown in Figure 3. When the dimensionless integrated meshing error value *E*_*spi*_^(1)^=  = 0.05, the system is in a single-cycle motion state, the time history graph is close to a sinusoidal curve, the vibration amplitude between cycles is basically the same, the phase trajectory line is an elliptical closed curve, the Poincaré diagram is a single point and the fundamental frequency signal in the spectrum is very prominent at this time, indicating that the system is in a typical single-cycle state.

The article "Nonlinear Dynamic Response Analysis of a Three-Stage Gear Train Based on Lightweight Calculation for Edge Equipment" was published in 2022. Journal: Comput Intell Neurosci.

With the increase of the integrated meshing error, when 0.779, as shown in Figure 4, the time course diagram changes periodically with two amplitudes as one cycle, the phase trajectory line is concave from one elliptic curve to two elliptic curves, the Poincaré cross-sectional diagram splits from one single point to two single points, and the FFT spectrum is shown as octave components, indicating that the system is in a two-cycle motion state. Combining Figures 3 and4, it can be found that the motion state of the system splits and changes from single-cycle to two-cycle and four-cycle with the increase of the magnitude of the integrated dimensionless mesh error. At the integrated dimensionless meshing error (1) *E*_*spi*_^(1)^= 1.259, strange attractors appear in the cross-sectional plot of Poincaré, indicating that the system enters the chaotic state through multi-cycle bifurcation at this time. When (1) *E*_*spi*_^(1)^ reaches 0.939, the system bifurcates from the two-cycle state to the two-cycle state with an LLE value of -0.001713. Therefore, the “negative pole” that appears in the plot of the maximum Lyapunov exponent of the system under the change of the integrated mesh error can characterize the dynamics of the two-cycle bifurcation, as shown in Figure 5.

## 7. Conclusion

In this paper, a modified stochastic regression method is used to solve a system of vibration differential equations for a three-stage gear train, and the effects of changes in the integrated dimensionless excitation frequency and the integrated meshing error on the dynamic response of the system are analyzed. A new static no-load transmission error model is established, which has its unique advantages in the fault diagnosis of gears. The model no longer requires tooth surface equations, avoiding the difficulty of merging tooth surface errors into tooth surface equations. The effect of the static unloaded transmission error of the real tooth surface on the dynamic characteristics of the bevel gear is analyzed. The model is also applicable to other types of gears. The global bifurcation diagram, Poncelet cross section diagram, and phase trajectory diagram are used as the main basis, and the time history diagram and the spectrum diagram are used as auxiliary tools to determine the range of bifurcation parameters when the three-stage gearing system is in a relatively stable state. It is found that the system is in a relatively stable state when the dimensionless excitation frequency is in the range of 0.716–0.86 and the magnitude of the dimensionless integrated meshing error is < 1.089.

The article "Nonlinear Dynamic Response Analysis of a Three-Stage Gear Train Based on Lightweight Calculation for Edge Equipment" was published in 2022. Journal: Comput Intell Neurosci.

## Figures and Tables

**Figure 1:** System under the variation of the integrated meshing error.

**Figure 2:** Plot of the maximum Lyapunov exponent of the system under the variation of the integrated error.

**Figure 3:** Dynamics of the system at *E* = 0.05.

**Figure 4:** Dynamics of the system at *E* = 0.779.

**Figure 5:** Dynamics of the system at *E* = 0.956.

**Table 1:** Basic parameters of a three-stage gear train.

		Planet carrier *C*	Sun wheel *S*	Planetary gear *p*	Inner ring gear *r*
*First stage planetary gear train(number of planetary gears N*_1_ *=* *3)*					
Radius of base circle Rb/(m)		0.471	0.196	0.243	0.683
Mass M/(kg)		2042.9	345.0	388.3	410.3
Moment of inertia im/(kg *m*^2^)		462.56	7.63	16.26	226.58
Average meshing stiffness kel/(n/M)		—		1.31 × 10^10^	1.49 × 10^10^
Stiffness variation amplitude kal/(n/M)		—		4.97 × 10^9^	5.12 × 10^9^

*First stage planetary gear train (number of planetary gears N*_2_ *=* *3)*					
Radius of base circle Rb/(m)		0.351	0.133	0.194	0.157
Mass M/(kg)		1212.6	132.4	176.6	81.6
Moment of inertia im/(kg *m*^2^)		151.76	1.30	5.13	26.66
Average meshing stiffness kel/(n/M)		—		2.62 ×10^10^	2.54 ×10^10^
Stiffness variation amplitude kal/(n/M)		—		7.54 ×10^9^	3.23 ×10^9^

## Data Availability

The data used to support the findings of this study are available from the corresponding author upon request.
